This article has been retracted.

# Design and Implementation of Balance Ability Assessment Training System for Special Children Based on Education Cloud Integration

**DOI:** 10.1155/2022/9359367

**Published:** 2022-09-26

**Authors:** Yan Lu, Mingming Xing, Jian Song

**Affiliations:** ^1^College of Education, Tongren University, Guizhou, China 554300; ^2^College of Material and Chemical Engineering, Tongren University, Guizhou, China 554300

## Abstract

Many children with special needs have body balance disorders, which will not only bring inconvenience to their daily lives but also have a certain impact on their spirits, making them insecure. It will lead to a decline in their social skills, which will also seriously affect their study and work as well as reduce their quality of life. The purpose of this paper is to design and discuss a system for evaluating and training the balance ability of children with special needs based on the integration of education cloud. The balance ability evaluation module of the system performs a series of calculations on the projection coordinates of the center of gravity of the human body in various postures, and the obtained parameter values are the basis of the evaluation. This paper analyzes the role of education cloud integration in the evaluation of balance ability of special children, evaluates and trains the balance ability of special children, and verifies the feasibility of the balance ability evaluation and training system for special children. This study found that in a feasibility trial evaluating the balance ability of children with special needs, the balance stability of the tested children was improved, and the overall balance ability improved by 60%. The balance ability evaluation training system developed in this paper can effectively improve the independent standing ability of young children. Children over the age of 4 do not have any difficulties in understanding and mastering movements, and training difficulties for children are also applicable. At the same time, the results of these exercises also showed that this kind of exercise can help children maintain their balance.

## 1. Introduction

The human body's ability to balance is the ability to maintain maximum stability in any situation and to be able to self-regulate and maintain stability in any situation. The balance ability of the human body means that no matter what posture the body is in, the body can maintain maximum stability and can self-regulate and maintain its own stability when it moves or is affected by external forces. That is to say, the body posture is maintained, and the body balance is maintained. It can flexibly adjust its own posture in any action, which can respond quickly and safely under the condition of external interference. Childhood is a critical period for human development, and maintaining a good balance is critical. Many children with special needs have the problem of balance dysfunction. The imbalance of balance function will not only affect their daily life but also have a profound impact on their psychology, making them insecure. This will lead to their inability to carry out normal interpersonal communication and even affect their future study and work, reducing their quality of life.

A very high proportion of children with special needs have balance disorders, and many are ignored because their balance disorders are not obvious. As the most basic function of many motor functions, balance function is very important to individuals. Without good balance ability, it will not only affect children's motor functions but also have a bad impact on children's psychology. Therefore, it is very important to pay attention to the development of children's balance ability and to carry out rehabilitation training in time when obstacles are found. This paper is aimed at designing and studying the evaluation and training system for the balance ability of special children based on the integration of education cloud, in order to make certain contributions to the balance ability of special children.

According to the research progress at home and abroad, different researchers have conducted corresponding collaborative research in the aspect of balance ability assessment training. The Wii Balance Board (WBB) is a commonly used balance assessment tool, but it needs to be clarified that the WBB has reported inconsistent validity when used to assess healthy young adults. Kaewkaen et al. explore the concurrent validity and reliability of the WBB in the assessment of balance in healthy young adults [1]. The purpose of Hamed et al.'s study was to evaluate the effectiveness of specific exercise interventions that control mechanisms of dynamic postural stability in older adults under unstable conditions [2]. The study by Oki et al. is aimed at identifying the main risk factors for falls in patients with Alzheimer's disease by comparing the balance, cognition, and visuospatial abilities of those who experienced falls and those who did not [3]. Krejci et al. aimed to analyze the interaction between levels of body balance, achievement of physical activity, anthropometric determinants, and psychosocial indices in older adults over the age of 65, in relation to gender and age [4]. The purpose of Vernadakis et al.'s study was to determine whether there are differences between an exercise game-based physical balance training program and a traditional adaptive physical balance training program in deaf adolescents [5]. However, these scholars' research on balance ability assessment training lacks technical proof. The research found that the research on balance ability evaluation and training based on education cloud integration has certain reliability, and the relevant literature on education cloud integration was consulted.

At present, some scholars have conducted in-depth research on the integration of education cloud: by exploring the relationship between cloud computing and the Internet of Things. Bijarbooneh et al. proposed a cloud-based solution that minimizes energy consumption by selecting sensors for sampling and relaying data, considering link quality and spatiotemporal correlation of data [6]. Kumar proposed a security technique for image fusion using mixed domains for privacy protection and copyright protection. The proposed method provides a secure technique for digital content in cloud environments [7]. It is necessary to improve the design of educational resource information sharing algorithm in cloud computing environment. Gao proposed an educational resource information sharing algorithm based on big data association mining and quasilinear regression analysis [8]. The main purpose of Choudhary was to explore various application fields of cloud computing and provide an overview of the fields of cloud computing usage. He discussed the key roles played by cloud computing in different fields [9]. Based on this, Zhang C. and Zhang X. designed and implemented a multimedia system based on the Internet of Things and cloud service platform based on the actual needs [10]. However, scholars at home and abroad have not conducted in-depth research on the design and implementation of the balance ability evaluation training system for special children on this basis but only unilaterally discussed its significance. On the basis of the integration of education cloud, this paper conducts experimental research on the design and implementation of the balance ability evaluation training system for special children.

Most balance assessment systems are suitable for adults and do not specifically consider some factors specific to children, such as children's poor tolerance and difficulty in control. The work done in this paper is to design and implement a system for special children, in order to screen the measurement postures that are easy for children to operate, the measurement parameters with better stability, and the algorithm to optimize the parameters. An accurate and objective quantitative assessment of its balance ability can be made. Through the analysis of various indicators, the results show that the overall balance stability of the subjects has been improved, and the overall balance has increased by 60%. This system can be used for training of young children who have reached independent standing. Children aged 4 and above can understand movements without obstacles, and the training difficulty is suitable for young children. The training effect also shows that this training has a certain promotion effect on the balance ability of the children.

The innovations of this paper are as follows: (1) the definition and advantages of cloud education are analyzed and discussed. (2) The balance ability assessment training system for special children is tested and optimized. (3) The feasibility of the special children's balance ability assessment training system for special children is tested.

## 2. Design and Implementation Method of Training System for Special Children

### 2.1. Cloud Education and Its Advantages

Cloud computing is a computing method, but its characteristics are based on the Internet. In this way, computers and other devices can provide common software, hardware, and information as needed. “Cloud” is a metaphor for the network and the Internet. Cloud education is a platform based on the idea of cloud computing, which uses cloud computing technology to allocate, manage, and share teaching resources to meet the needs of modern teaching methods and personalized learning [11]. Cloud teaching breaks through the boundaries of traditional education informatization and proposes a new concept of teaching informatization. Teachers and students only need one account to log in to the cloud teaching platform through the account. They can obtain resources. Cloud teaching can effectively overcome the current teaching environment and solve the problem of low level of educational informatization [12]. Cloud education technology effectively connects terminals around the world through the network, so that educators and students can obtain high-quality educational resources from the cloud. At the same time, it can also upload high-quality resources in its hands to the cloud and collaborate in the cloud to jointly develop high-quality educational resources.  Figure 1 shows the operation mode of the cloud education platform.

Therefore, the biggest function of cloud education is to share educational resources regardless of region, person, time, region, or time and realize the sharing of educational resources in the three major systems of school education, family education, and social education. At the same time, it also provides a new education method for mobile learning, blended learning, flipped classroom, etc.

Cloud education platform is a brand-new information teaching environment, which enables learning resources to be shared everywhere through cloud services, thus promoting the large-scale application of mobile learning. The cloud education platform not only has some basic functions of the traditional online teaching platform but also has its own advantages [13].

#### 2.1.1. Providing “One-Stop” Service

Cloud education platform integrates teaching, management, communication, and other teaching services. Using portal technology, users can enjoy one-time login and cross-site access one-stop service with only one account [14]. The virtual learning environment cloud education platform provides learners with a variety of learning functions. After logging in, users can click on different functional modules according to their own preferences to enter the corresponding learning scene and conduct on-demand learning [15].

#### 2.1.2. Fully Sharing Educational Resources

Cloud education stores resources in the cloud, allowing users to upload resources to the cloud at any time and download resources freely, so as to achieve resource sharing based on people, topics, and types. Supporting multiple interactions, through the cloud teaching platform, it can realize multilevel interactions such as family, school, and society. It can realize the deep interaction of homework, information, and ideas, allowing learners to share learning experience and achieve cooperative learning goals [16].

#### 2.1.3. Ubiquity of Learning

The cloud education platform covers the main learning locations of students and realizes the generalization of the learning environment. Students log in to the cloud teaching platform through their mobile phones to obtain learning resources and participate in learning, which makes learning not be limited by geographical location and can be achieved in real time [17].

### 2.2. Role of Education Cloud Integration in the Evaluation of Balance Ability of Special Children

Good balance is essential to people's daily lives. Various basic activities of the human body, such as sitting, standing, walking, dressing, and eating, are based on a good balance function. The development of balance ability can enhance the function of motor organs and the function of vestibular organs, thus improving the regulation effect of the central nervous system on muscles and internal organs. It can also promote the activities of the body, enhance the adaptability to complex environments, and enhance its self-defense ability. Balance dysfunction will not only affect the normal activities of the body but also cause inconvenience to people's life and study. When children are in the process of growth, the cultivation of balance ability is conducive to children's perception of uprightness, direction, and distance, which lays the foundation for children's spatial perception. Children's balance dysfunction can lead to unsteady standing, sitting still, restless, falling easily, and insecure, which seriously affects their interpersonal relationships and also affects their study and work, reducing their quality of life [18–20]. Many special children have body balance disorders. For some children, such as those with cerebral palsy and paediatric palsy, abnormalities in their balance function can be directly observed. There are also children, such as children with hearing impairment, autism, ADHD, inattention, and sensory integration disorders, whose balance dysfunction is not obvious or does not significantly affect their daily life, which is often ignored. The training of balance ability has not been popularized in many special schools. However, abnormal balance function will affect the overall motor function of the individual. For example, it is easy to fall during sports activities, and it is impossible or difficult to perform activities that normal children can perform. These conditions, in turn, can have a serious impact on their life and learning. Therefore, accurate assessment and appropriate training of the balance ability of these special children are crucial for their physical and mental development [21].

The construction of “cloud computing” in the education sector will greatly promote information sharing, infrastructure construction, and campus information management. The value of cloud computing lies in its flexibility, scalability, and high performance ratio. It has the advantages of virtualization, dynamic scalability, and high reliability. First, cloud computing can build a unified information platform for schools. Second, it can effectively integrate all kinds of information on campus. Third, cloud computing can connect many information systems on campus to each other. Ultimately, cloud computing could allow schools to make better use of these infrastructures. Therefore, it is very reasonable to move the new computing model of cloud computing to the field of education to form an education cloud. This paper is aimed at designing and discussing the evaluation and training system for the balance ability of special children based on the integration of education cloud. The balance ability evaluation and training system for special children studied in this paper is also constructed based on the cloud computing education platform. Firstly, the training of children's balance ability is simulated and analyzed through cloud computing, and the optimal training mode is obtained, which is then applied to children [22].

### 2.3. Design of Balance Ability Assessment Training System for Special Children

#### 2.3.1. Determination of Data Collection Plan

The balance ability evaluation training system for special children is based on the pressure plate technology, which collects the distribution of human body gravity through the pressure sensor and transmits the data to the computer. Then, the position of the projection of the center of gravity of the human body is calculated by the computer software. The trajectory of the projection of the center of gravity is drawn, and a series of parameters of the projected trajectory of the center of gravity are calculated to understand the balance ability of the subject.

Four pressure sensors are used to collect human pressure values. If the number of selected sensors is small, such as two, the balance of the human body can only be judged in one direction. If the number of sensors is large, the shape and size of the subject's feet will be limited. Four pressure sensors correspond to the forefoot and rear heel of the two feet, which can judge the front-to-back balance ability and left-right balance ability of the human body, as well as other inclination directions of the human body. Therefore, four sensors are used for data collection. The sensor placement position corresponds to an included angle of 30° between the two feet, and the diameter of the contact surface of each sensor is 70 mm. After fixing the cover, the error caused by the changing moment of the foot size can be reduced.

The design of the evaluation module mainly includes screening evaluation parameters and screening evaluation posture. The balance ability evaluation module of the system performs a series of calculations on the projection coordinates of the center of gravity of the human body in various postures, and the obtained parameter values are the basis of the evaluation. Therefore, it is necessary to select or add evaluation indicators according to the characteristics and needs of young children and to design a relatively stable evaluation model.

#### 2.3.2. Implementation of the Evaluation Module

*(1) Barycentric Projection Coordinate Method*. The parameter calculation is based on the coordinates of the barycentric projection, so the calculation of the barycentric projection coordinates should be performed first.

Assuming that the coordinate plane is the force plane of the pressure sensor (parallel to the horizontal plane) and the origin is the standard barycentric coordinate point, the coordinates of the four pressure sensors are *X*(*i*_1_, *j*_1_), *Y*(*i*_2_, *j*_2_), *Z*(*i*_3_, *j*_3_), and *W*(*i*_4_, *j*_4_), respectively. The origin is *R*(*I*, *J*); *k*_1_, *k*_2_, *k*_3_, and *k*_4_ are the pressures of the four sensors.

The body gravity *G* is

(1) $$\begin{array}{c} G=\sum k_{n}=k_{1}+k_{2}+k_{3}+k_{4}. \end{array}$$

According to the principle of moment balance, the moment in direction *i* and direction *j* can be obtained as

(2) $$\begin{array}{c} Q_{i}=\sum k_{n}i_{n}=k_{1}i_{1}+k_{2}i_{2}+k_{3}i_{3}+k_{4}i_{4}, \end{array}$$

(3) $$\begin{array}{c} Q_{j}=\sum k_{n}j_{n}=k_{1}j_{1}+k_{2}j_{2}+k_{3}j_{3}+k_{4}j_{4}. \end{array}$$

The coordinates to calculate the actual barycentric projection are expressed as

(4) $$\begin{array}{c} I_{v}=\frac{Q_{i}}{G}=\frac{\left(k_{1}i_{1}+k_{2}i_{2}+k_{3}i_{3}+k_{4}i_{4}\right)}{\left(k_{1}+k_{2}+k_{3}+k_{4}\right)}, \end{array}$$

(5) $$\begin{array}{c} J_{v}=\frac{Q_{j}}{G}=\frac{\left(k_{1}j_{1}+k_{2}j_{2}+k_{3}j_{3}+k_{4}j_{4}\right)}{\left(k_{1}+k_{2}+k_{3}+k_{4}\right)}. \end{array}$$

*(2) Calculation Process*. After the upper computer detects the USB communication connection with the lower computer, it waits for the start detection command. When the subject stands on the balance table and is ready, the operator selects the test time and posture and clicks start. Then, the evaluation begins.

First, preparatory work such as initialization is performed. The parameter calculation thread is started, and the timing is started.

The frequency of the body's center of gravity shaking is about 1 ~ 1.5 Hz, and the selected sampling rate is 20 Hz, which is enough to accurately describe the real center of gravity shaking. Therefore, data is selected from the lower computer every 50 ms. At this time, the voltage value read in hexadecimal system is converted into decimal number first. The voltage value in decimal system is obtained as Vol (V), and the voltage value is converted into weight value *Q* (kg). The sensor range used is 0-75 kg. Under the output voltage of 0 ~ 5 V, the A/D chip used has a conversion accuracy of 12 bits. The calculation formula of the obtained weight value is

(6) $$\begin{array}{c} Q=\frac{\text{Vol}}{5}*75. \end{array}$$

The voltage accuracy *v* is

(7) $$\begin{array}{c} v=\frac{V}{4096}=1.2\text{ mV}. \end{array}$$

The measurement weight accuracy *q* is

(8) $$\begin{array}{c} q=\frac{75\text{ kg}}{4096}=0.02\text{ kg}. \end{array}$$

The effective value of 4 points of pressure is obtained from the lower computer, and the coordinate value of the projection of the center of gravity is calculated and displayed. The pressure value data obtained from each sampling is written to a file for backup. In order to improve the speed, the instantaneous intermediate values used in the formula, such as the instantaneous angle of the horizontal and vertical coordinates, are calculated at the same time. When the test time is over, the final value of each parameter is calculated and stored in the database.

## 3. Experiment Results of Design of Balance Ability Assessment Training System

### 3.1. Detection and Optimization of Balance Ability Assessment Training System

There are many ways to check the balance function, which can be roughly divided into two categories: static balance and dynamic balance. The balance function detection training system mainly uses the pressure values generated by the four focus points of the two soles of the human body on the sensor when the human body is standing and then measures the movement of the coordinates of the center of gravity of the human body through an algorithm. The measured pressure value directly affects the accuracy of the center of gravity coordinates, thereby affecting the test results.

Testing purpose: the error of the pressure value collected by the host computer and the error of the coordinates calculated by the program are measured. The cause of the error is analyzed, adjusted, and optimized to reduce the error

Testing tools: 4 pieces of standard broken code 5 kg, 10 kg, and 15 kg

Testing object: the evaluation module of the balance ability evaluation training system for special children. The test data is the final pressure value collected by the system and the calculated coordinate value

Testing method: the balance ability evaluation training system for special children starts from measuring the pressure value with the sensor to outputting the coordinates of the center of gravity. The process is shown in Figure 2

Among them, the generated system hardware errors, including the error of the pressure sensor itself, the sampling, and quantization of data, that is, the error from analog to digital and the error generated during data transmission, are mostly random errors. The purpose of error analysis is to verify the accuracy of the pressure output value and barycentric coordinates, as well as to analyze the position and correction method of the main error.

In this paper, the standard weights with the sum of the four weights that are closer to the children's weight range are selected as 5 kg, 10 kg, and 15 kg for the combined test, and the combined weight range is between 20 kg and 45 kg. The center position and the coordinates of the eight directions of front, rear, left, right, front left, front right, rear left, and rear right are measured, respectively.

The relative error of the four-way pressure value calculated from the first measurement value is analyzed, and the line graph is drawn as shown in Figure 3. It can be seen from the line graph that the measured values of pressure signal 1 and pressure signal 4 are generally too large, and the relative deviation does not exceed 7.2%. The measured values of pressure signal 2 and pressure signal 3 are generally small, and the relative deviation does not exceed 16.6%.

The mean and standard deviation of the relative errors of the four pressure signals are shown in Table 1.

The error analysis is carried out on the calculated coordinates of the first measurement value, as shown in Figure 4. Among them, the *X* coordinate error range is between -6 mm and 6 mm, and most of the error values are distributed around -2 mm. The average value of the calculated *X*-sitting error is -1.928 mm. The standard deviation is 2.421 mm, and the maximum value is 5.63 mm. That is to say, the measured value is to the left of the visual perception than the theoretical value. The *Y* coordinate error range is between -6 mm and 4 mm, and most of the error values are distributed between -1 mm and 1 mm. The *Y* seat cup error has an average value of -0.791 mm, a standard deviation of 1.912 mm, and a maximum value of 5.207 mm.

According to the above error measurement results, the four pressure signals have a relatively obvious deviation trend, and software calibration can be performed. The measurement system is decided to be optimized as follows: first, the pressure signal measurement value is calibrated by the software, and a coefficient of the relative error average is subtracted from the four pressure signals. That is, the original data is multiplied by (1 − *A*), and *A* is the relative error average. Second, the random error is reduced by taking the average value of multiple samples. That is, for each time, 5 groups of data in the sampling area of the pressure value are calculated, and the average value of the 5 groups of data is calculated as the effective value of this data collection.

After optimization, the same measurement method is used for the second measurement, and the relative error of the four pressure values is calculated, as shown in Figure 5. The relative error range of the final four pressure value is between -5.6% and 3.8%, which is a great improvement over that before optimization.

Through the calculation, the standard value of the relative error of the calculated four-way pressure value is shown in Table 2. It can be seen from the error mean that compared with the first error mean, there is a great improvement.

After optimizing and improving the measured value of the pressure signal, the coordinate error of the second measurement is obtained as shown in Figure 6.

The mean value of the calculated *X*-coordinate error is -0.634 mm. The standard deviation is 0.931 mm, and the maximum value is 1.70 mm. The average value of the *Y* coordinate error is -0.498 mm. The standard deviation is 0.779 mm, and the maximum value is 1.72 mm. It can be seen from the line chart that the second measurement error is significantly improved compared to the first measurement error, which meets the test requirements.

### 3.2. Feasibility Test of the Balance Ability Assessment Training System for Special Children

This paper designs and implements a training system for evaluating balance ability. Because it applies to children with special needs, whether the operation rules of the training game are easy to understand and whether the training difficulty is operable directly affect the training effect. It is very necessary to carry out game training for the balance ability evaluation training system of special children. Therefore, this paper verifies the feasibility of the system training module.

The subject of this experiment was a 4-year-old male child. The child suffered from cerebral palsy and hearing impairment, who had normal intelligence. His balance ability could reach the level of autonomous standing. When standing, his body would sway from side to side and could not maintain long-term stability in one position.

In view of the subject's own situation, this paper first selected the “collect carrots” game to train him. Before training, his balance ability was evaluated. Because the purpose of this experiment was to verify the feasibility of the training game, only one posture of standing on a solid surface was performed. Because each assessment of the subjects was compared with themselves, it was not necessary to analyze the two parameters of the trajectory length per unit height and the trajectory length per unit weight.

During the training process, the boy stood on the balance table and used the shaking of the body to change the position of his center of gravity to complete the tasks required by the training game. If it was difficult for him to complete, he could hold the railings to complete but tried to ask the subjects not to rely too much on the railings.

For the boy's training, if he had been trained in one way, his interest would be weakened, and he might be negatively trained. Therefore, in this experiment, the training process was divided into 5 sections, and the training content of each section is shown in Table 3. Each session lasted roughly 7 minutes, with a 3-minute rest between each session, followed by an assessment. The entire training process lasted about an hour, with a total of 5 training sessions.

The rehabilitation tracking module of the system records the evaluation data before training and after 5 training sessions.

Figure 7 shows the variation trends of the *X*-direction trajectory length and the *X*-direction trajectory mean square error before and after 5 training sessions. The abscissa represents the number of training sessions. Both parameters represent the balance ability of the subject in the left and right directions. Since the first and second stages mainly train the subject's ability to keep their balance by leaning left and right, the *X*-direction trajectory length has a more obvious downward trend after two left and right balance training. The performance trend of the mean square error in the *X*-direction is not very obvious, and there will be a more significant improvement after a longer period of training.

Figure 8 shows the trend of *Y*-direction trajectory length and *Y*-direction trajectory mean square error before and after 5 training sessions. The abscissa represents the number of training sessions. Both parameters represent the balance ability of the subjects in the left and right directions. Since the third and fourth stages mainly train the subject's ability to maintain balance by leaning forward and backward, the *Y*-direction trajectory length has a more obvious downward trend after two front and rear balance training. The performance trend of the mean square error in the *Y*-direction is not very obvious, and there will be a more significant improvement after a longer period of training. Through the analysis of the above parameters, it can be seen that the stability of the children's finishing balance has been improved, and the overall balance can be improved by 60%.

Combined with the above experimental results, it is shown that the balance ability evaluation training system designed in this paper can cultivate children's independent standing ability. Children 4 years old and above have no obstacles in understanding the training operation, and the training difficulty is suitable for children. At the same time, the results of the training also showed that such exercises help children's balance. This system is suitable for children with special needs to carry out game training.

## 4. Conclusion

The role of cloud computing in education is not only in terms of learning but also in the convenience of campus life. An education cloud platform has been built, and a smart campus has been built to ensure the interoperability of all data. It can not only meet the characteristics of interaction and personalization in the network environment but also adapt to the new educational informatization needs, achieve maximum sharing, and prevent the repeated use of educational systems and waste of resources. Based on the integration of education cloud, this paper discusses the balance ability evaluation and training system for children with special needs. Using the balance ability assessment training system developed in this paper, a child with cerebral palsy with hearing impairment was trained for balance ability. Assessments of balance ability before and after each exercise showed that the child's overall balance ability improved. Combined with the subjective observation of the testers in the experiment, the subject who need to hold the handrail for training at the beginning do not need to hold the handrail at the end, which can show that the problem of their balance disorder has improved. The above experiments show that the system can train children who have reached the level of autonomous standing. Children aged 4 and above have no obstacles in understanding the content of the training operation, and the difficulty of training is also suitable for children. The training results also show that this training is helpful for children's balance ability to a certain extent. Therefore, the system is suitable for game training of special children. This paper will build an intelligent decision-making system in the follow-up to realize the intelligent connection between evaluation and training. According to the different evaluation results, it can intelligently provide training content and can provide training assistance for the trainer.

## Figures and Tables

**Figure 1:** Operation mode of cloud education platform.

**Figure 2:** Error analysis flow chart.

**Figure 3:** Line chart of relative error of pressure signal.

**Figure 4:** *X* and *Y* coordinate errors of the first measurement.

**Figure 5:** Relative error of the second measurement pressure value.

**Figure 6:** *X* and *Y* coordinate errors of the second measurement.

**Figure 7:** Test value of *X*-direction trajectory length and trajectory contrast test value before training and after 5 times of training.

**Figure 8:** *Y*-direction mean squared error test values before training and after 5 training sessions.

**Table 1:** Mean and standard deviation of the error of the first measurement of the pressure signal.

Pressure signal	Average value	Standard deviation
1	0.024	0.046
2	-0.076	0.046
3	-0.094	0.036
4	0.035	0.019

**Table 2:** Mean and standard deviation of the error of the second measurement of the pressure signal.

Pressure signal	1	2
Average value	-0.003	0.009

Pressure signal	3	4
Average value	-0.012	-0.004

**Table 3:** Training program.

Numbering	Training phase	Training content
1	The first stage	Collect carrots (special training in left and right directions)
2	Second stage	Collect carrots (special training in left and right directions)
3	The third phase	Collect carrots (special training in front and rear directions)
4	Fourth stage	Collect carrots (special training in front and rear directions)
5	The fifth stage	Collect carrots (integrated training)

## Data Availability

The data used to support the findings of this study are available from the corresponding author upon request.
